The article "Clinical Effect of Laparoscopic Radical Surgery Combined with Neoadjuvant Chemotherapy in Treating Cervical Cancer and Its Influence on Postoperative Complications and Adverse Reaction Rates" was published in 2022. Journal: J Healthc Eng.

# Clinical Effect of Laparoscopic Radical Surgery Combined with Neoadjuvant Chemotherapy in Treating Cervical Cancer and Its Influence on Postoperative Complications and Adverse Reaction Rates

**DOI:** 10.1155/2022/8768188

**Published:** 2022-02-09

**Authors:** Wenduan Gong, Yejun Liu

**Affiliations:** Department of Gynecology, Qianjiang Central Hospital of Hubei Province, Qianjiang 433100, Hubei, China

## Abstract

**Background:**

Cervical cancer, the only gynecological malignancy for which a clear pathogeny has been established, has an incidence rate only second to breast cancer.

**Objective:**

In our study, we aim to investigate the clinical effect of laparoscopic radical surgery combined with neoadjuvant chemotherapy in treating cervical cancer and its influence on postoperative complications and adverse reaction rates.

**Methods:**

Cervical cancer patients admitted to our hospital from August 2018 to May 2020 were retrospectively analyzed as the research object and divided into the control group and the experimental group by the draw method, with 50 cases in each group. The laparoscopic radical surgery was performed on the control group, and the laparoscopic radical surgery combined with neoadjuvant chemotherapy was performed on the experimental group to compare their effective rates, adverse reaction rates, postoperative complication rates, expression levels of serum tumor necrosis factor-*α* (TNF-*α*) and soluble interleukin-2 receptor (SIL-2R) inside the body before surgery and at one week after surgery, quality of life (QLI) scores, and Mental Status Scale in Nonpsychiatric Settings (MSSNS) scores.

**Results:**

Compared with the control group, the experimental group obtained significantly higher effective rate and QLI scores (*P* < 0.05) and significantly lower adverse reaction rates, postoperative complication rates, expression levels of serum TNF-*α* and SIL-2R inside the body at one week after surgery, and MSSNS scores (*P* < 0.05), with statistical differences; before surgery, the TNF-*α* and SIL-2R expression levels of the two groups were not significantly different (*P* > 0.05), but the levels at one week after surgery were significantly lower than those before, indicating statistical significance (*P* < 0.05).

**Conclusion:**

The clinical effect of laparoscopic radical surgery combined with neoadjuvant chemotherapy can obviously improve the effective rate of cervical cancer patients and lower the incidence rates of postoperative complications and adverse reactions.

## 1. Introduction

Cervical cancer is a common malignant tumor in the female reproductive system characterized by high mortality and recurrence rate, but usually, no specific clinical manifestations occur before the onset of the disease, so patients are tending to ignore some minor abnormal situation of the body and thus miss the optimal treatment time [1–3]. Women over the age of 45 are the usual and vulnerable victims of cervical cancer. However, with the changes in people's lifestyles recently, more and more younger women are diagnosed with cervical cancer. Currently, the most common clinical treatment for the disease is surgery, namely, performing tumor tissue resection to prevent the tumor cell diffusion and then achieve the curative effect [4–6]. Traditionally, the resection of tumor tissue is conducted by laparotomy, but such a surgical method poses a great impact on the patients and slows down the recovery process and even causes some serious complications. With the progress of scientific technology and medical technology, minimally invasive techniques have been applied widely in medical work, and so has laparoscopic surgery [7–9]. Neoadjuvant chemotherapy is the chemotherapy pattern performed before surgery in patients with advanced malignant tumors, which shrinks the tumor, downs the tumor stage, decreases the surgical difficulty, and increases the success rate [10–12]. Cervical cancer, the only gynecological malignancy for which a clear pathogeny has been established, has an incidence rate only second to breast cancer. The incidence of cervical cancer is closely related to the times of giving birth, health habit, living habit, and the time of first sex, and the disease can be classified as squamous cell carcinoma, adenocarcinoma, adenosquamous carcinoma, etc., with the main manifestations such as vaginal bleeding, vaginal pain, and anemia [13–15].

Thus, we aim to explore the curative effect of laparoscopic radical surgery combined with neoadjuvant chemotherapy in treating cervical cancer patients and analyze its influence on postoperative complications and adverse reaction rates. And we chose cervical cancer patients as the research object for the study and performed the laparoscopic radical surgery alone as well as the combined treatment, respectively, to the two groups to compare the effective rates, adverse reaction rates, postoperative complication rates, expression levels of intracorporal serum TNF-*α* and SIL-2R before surgery and at one week after surgery, quality of life (QLI) scores, and Mental Status Scale in Nonpsychiatric Settings (MSSNS) scores, with the specific study reported as follows.

## 2. Materials and Methods

### 2.1. General Information

The cervical cancer patients admitted to our hospital from August 2018 to May 2020 were retrospectively analyzed as the research object and divided into the control group (40–78 years old) and the experimental group (38–75 years old) by the draw method, with 50 cases in each group. The general information such as the age of patients in both groups was not significantly different, with no statistical significance (*P* > 0.05) (see Table 1).

### 2.2. Inclusion/Exclusion Criteria

#### 2.2.1. Inclusion Criteria

The inclusion criteria were defined as follows:

1. The patients who met the clinical signs of cervical cancer
2. The patients who were 18 years old or older
3. The patients who had no drug abuse history, drug allergy history, or bad addictions
4. The patients who were conscious and able to cooperate with the study with normal mental status
5. The study was approved by the Hospital Ethics Committee, and the patients joined the study voluntarily by signing the informed consent.

#### 2.2.2. Exclusion Criteria

The exclusion criteria were defined as follows:

1. The patients who were recently treated with anticoagulant medication and had coagulation disorder
2. The patients who had other organic diseases or malignant tumors
3. The patients who were recently treated with anesthetic drugs or other surgeries
4. The patients whose clinical information was insufficient

### 2.3. Methods

The patients in the control group were given laparoscopic radical surgery with the following specific steps. The modified bladder lithotomy position was taken and a cushion was put under the buttocks of the patient, an incision was made at 4 cm away from the upper edge of the nabhi chakra, the casing needle was inserted to establish the pneumoperitoneum, the intraabdominal pressure was maintained between 12 and 15 mmHg, the laparoscopy was inserted to observe the abdominal cavity and the pelvic cavity, and the hysterectomy was performed according to the image displayed by the laparoscopy; after surgery, the wound was rinsed, sutured, disinfected, and bound up [16–18].

Before the aforesaid surgery, the patients in the experimental group were given neoadjuvant chemotherapy with the following specific steps. The chemotherapy was conducted once every three weeks and lasted for 3 days each time; between the two times of chemotherapy, routine physical examination was performed to the patients, and the administration was adjusted according to the conditions of the patients; after 2 courses of therapy, the same laparoscopic radical surgery as the control group was conducted.

### 2.4. Observation Indicators

The effective rates, adverse reaction rates, postoperative complication rates, expression levels of intracorporal serum TNF-*α* and SIL-2R before surgery and at one week after surgery, QLI scores, and MSSNS scores of the patients in the two groups were compared.

It was considered markedly effective if the clinical manifestations were basically disappeared, the tumor tissues were excised successfully, and no postoperative complications occurred; it was considered effective if the clinical manifestations were obviously alleviated, the tumor tissues were excised successfully, and mild postoperative adverse reactions occurred; and it was considered ineffective if the clinical manifestations were not obviously alleviated, the tumor tissues were not excised successfully, and severe postoperative reverse reactions occurred.

The scoring standards of the QLI scores included daily activities, work and life, and interpersonal relationship, and the maximum score of each standard was 10 points, with higher points indicating better QLI, and vice versa.

The MSSNS scores took 60 points as the dividing line, namely, less than 60 points indicated normal mental status, 60–70 points indicated mildly abnormal mental status, and over 70 points indicated abnormal mental status.

### 2.5. Statistical Processing

In this study, the data processing software was SPSS20.0, the picture drawing software was GraphPad Prism 7 (GraphPad Software, San Diego, USA), items included were enumeration data and measurement data, which were expressed as (*n*(%)) and (±*s*) and examined by *X*^2^ test and *t*-test, respectively, and differences were considered statistically significant at *P* < 0.05.

## 3. Results

### 3.1. Comparison of Effective Rates

The experimental group obtained a significantly higher effective rate than the control group, which was statistically different (*P* < 0.05) (see Figure 1).

### 3.2. Comparison of Complication Rates

The experimental group obtained a significant postoperative complication rate than the control group, which was statistically different (*P* < 0.05) (see Table 2).

### 3.3. Comparison of Adverse Reaction Rates

The adverse reactions occurred during treatment mainly included alopecia, frequent urination, hypodynamia, and nausea, and the adverse reaction rate of the experimental group was clearly lower than that of the control group, which was statistically different (*P* < 0.05) (see Figure 2). We can clearly see that figure A indicated the adverse reaction occurred in the experimental group, of which 3 cases had alopecia, 1 case had frequent urination, 1 case had hypodynamia, 2 cases had nausea, and the total adverse reaction rate was 14%. And figure B indicated the adverse reaction occurred in the control group, of which 5 cases had alopecia, 3 cases had frequent urination, 4 cases had hypodynamia, 4 cases had nausea, and the total adverse reaction rate was 32%.

### 3.4. Comparison of Expression Levels of Intracorporal Serum TNF-*α* and SIL-2R before Surgery with Those at One Week after Surgery

The result of comparing the expression levels before surgery was not statistically significant (*P* > 0.05), and at one week after surgery, the expression levels were obviously reduced, and those of the experimental group were clearly lower than those of the control group, with statistical significance (*P* < 0.05) (see Figures 3 and 4). From Figure 3, we can clearly see that the TNF-*α* expression levels before surgery and at one week after surgery of the experimental group were (2.86 ± 0.55) and (1.35 ± 0.41), respectively, and those of the control group were (2.85 ± 0.55) and (2.13 ± 0.47), respectively. Furthermore, Figure 4 shows that the SIL-2R expression levels before surgery and at one week after surgery of the experimental group were (598.33 ± 114.91) and (237.00 ± 56.43), respectively, and those of the control group were (600.82 ± 115.37) and (361.24 ± 70.00), respectively.

### 3.5. Comparison of QLI Scores and MSSNS Scores

Compared with the control group, the experimental group had obviously higher QLI scores and MSSNS scores, with statistical differences (*P* < 0.05) (see Figure 5).

## 4. Discussion

The main treatment for patients with cervical cancer is surgery, and laparoscopic radical surgery is commonly adopted in the clinic to remove the tumor tissue by minimally invasive techniques, thereby achieving the therapeutic effect. However, the surgical risk is greater and the success rate is smaller if cervical cancer reaches middle and advanced stages, so downstaging the tumor by narrowing the tumor tissue with the aid of certain adjuvant therapies is required [19–21]. Neoadjuvant chemotherapy refers to the chemotherapy for downstaging before the cervical cancer surgery, and it was reported that the combination treatment of neoadjuvant chemotherapy and laparoscopic radical surgery can remarkably improve the curative effect and lower the risk of postoperative complications [22–24]. Therefore, cervical patients were selected for the study, and the laparoscopic radical surgery alone and the combination treatment were, respectively, performed different groups to compare their effective rates, adverse reaction rates, postoperative reaction rates, expression levels of intracorporal serum TNF-*α* and SIL-2R before surgery and at one week after surgery, QLI scores, and MSSNS scores, thus exploring the clinical effect of the combination treatment and its influence on the postoperative complications and adverse reaction rates. Qi Qingxia and other scholars [25] pointed out in their experiment that neoadjuvant chemotherapy combined with laparoscopic radical surgery worked better in treating advanced cervical cancer patients, with fewer postoperative complications, which was consistent with the study and proved that the study results were scientific and reliable.

The study results showed that the effective rate and QLI scores of the experimental group were significantly higher than those of the control group, which were statistically significant (*P* < 0.05) and indicated that after the neoadjuvant chemotherapy, the laparoscopic radical surgery achieved a higher success rate and clinical effect. As the neoadjuvant chemotherapy was performed before the surgery, the tumor tissue was shrunk with the aid of chemotherapy, so a smaller range was required to be excised during surgery, which could not only save the operation time but also lower the possibility of relapse after surgery. In addition, compared with the control group, the experimental group obtained significantly lower adverse reaction rates, postoperative complication rates, expression levels of intracorporal serum TNF-*α* and SIL-2R at one week after surgery, and MSSNS scores, with statistically significance (*P* < 0.05); before surgery, the results of comparing the expression levels between the two groups had no statistical meaning (*P* > 0.05); and at one week after surgery, the expression levels were obviously lowered, presenting statistical differences (*P*< 0.05). The tumor necrosis factor-*α* (TNF-*α*) and soluble interleukin-2 receptor (SIL-2R) are targeted markers commonly used in the clinic to diagnose and treat malignancies, and the higher the expression levels of serum TNF-*α* and SIL-2R, the higher the stage of cancer, and vice versa. The above results showed that the expression levels of serum TNF-*α* and SIL-2R inside the body of patients undergoing neoadjuvant chemotherapy before laparoscopic radical surgery were significantly reduced, to the extent greater than the patients undergoing the laparoscopic radical surgery only; meanwhile, patients in the experimental group obtained significantly smaller incidence rates of adverse reactions and postoperative complications, indicating that the combination treatment was safer and posed less impact on the patients.

## 5. Conclusion

To sum up, the combined treatment of neoadjuvant chemotherapy and laparoscopic radical surgery can clearly improve the treatment effect of cervical cancer and lower the incidence rates of postoperative complications and adverse reactions, with a higher clinical value. Our finding is worthy of promotion and application in the clinic. Moreover, our study has obtained consistent results with other relative studies, which implies that our results are scientific and reliable. However, there are still some limitations in our study. We need to collect more data and conduct detailed data analysis.

## Figures and Tables

**Figure 1:** Comparison of effective rates. *Note.* Image A indicates the treatment efficacy of the experimental group, of which 27 cases were markedly effective, 17 cases were effective, 6 cases were ineffective, and the total effective rate was 88%; Image B indicates the treatment efficacy of the control group, of which 18 cases were markedly effective, 15 cases were effective, 17 cases were ineffective, and the total effective rate was 66%; and ^*∗*^indicates that the result of comparing the effective rates between the two groups was statistically significant (*X*^2^ = 6.83; *P* = 0.009).

**Figure 2:** Comparison of adverse reaction rates. *Note.*^*∗*^indicates that the result of comparing the adverse reaction rates between the two groups was statistically significant (*X*^2^ = 4.57; *P* = 0.03).

**Figure 3:** Comparison of TNF-*α* expression levels before surgery and at one week after surgery between the two groups. *Note.* The horizontal axis indicates before surgery and a week after surgery, and the vertical axis indicates the TNF-*α* expression levels in ng/ml. ^*∗*^ indicates that the results of comparing the TNF-*α* expression levels before surgery between the two groups were not statistically significant (*t* = 0.09; *P* = 0.93); ^*∗∗*^indicates that the results of comparing the TNF-*α* expression levels at one week after surgery between the two groups were statistically significant (*t* = 8.84; *P* < 0.001); ^*∗∗∗*^ indicates that the results of comparing the TNF-*α* expression levels before surgery with those at one week after surgery of the experimental group were statistically significant (*t* = 15.56; *P* < 0.001); and ^*∗∗∗∗*^ indicates that the results of comparing the TNF-*α* expression levels before surgery with those at one week after surgery of the control group were statistically significant (*t* = 7.04; *P* < 0.001).

**Figure 4:** Comparison of SIL-2R expression levels before surgery and at one week after surgery between the two groups. *Note.* The horizontal axis indicates before surgery and a week after surgery, and the vertical axis indicates the SIL-2R expression levels in pg/ml. ^*∗*^ indicates that the results of comparing the SIL-2R expression levels before surgery between the two groups were not statistically significant (*t* = 0.11; *P* = 0.91); ^*∗∗*^ indicates that the results of comparing the SIL-2R expression levels at one week after surgery between the two groups were statistically significant (*t* = 12.55; *P* < 0.001); ^*∗∗∗*^ indicates that the results of comparing the SIL-2R expression levels before surgery with those at one week after surgery of the experimental group were statistically significant (*t* = 19.96; *P* < 0.001); and ^*∗∗∗∗*^indicates that the results of comparing the SIL-2R expression levels before surgery with those at one week after surgery of the control group were statistically significant (*t* = 9.77; *P* < 0.001).

**Figure 5:** Comparison of QLI scores and MSSNS scores. *Note.* The horizontal axis from left to right indicates QLI and MSSNS, and the vertical axis indicates the scores (points); ^*∗*^ indicates that the QLI scores of the experimental group and the control group were (71.53 ± 9.46) and (64.18 ± 7.66), respectively, and the comparison results were statistically significant (*t* = 4.27; *P* < 0.001); and ^*∗∗*^ indicates that the MSSNS scores of the experimental group and the control group were (42.21 ± 3.38) and (48.01 ± 4.31), respectively, and the comparison results were statistically significant (*t* = 7.49; *P* < 0.001).

**Table 1:** Comparison and statistics of general information (±*s*, *n*).

Group	Experimental group	Control group	t/*X*^2^	*P*
Age (years)	59.86 ± 6.44	60.21 ± 6.71	0.27	0.79
Height (cm)	163.32 ± 5.80	162.59 ± 4.99	0.67	0.50
Weight (kg)	67.31 ± 10.25	67.71 ± 10.35	0.19	0.85
Duration of disease (months)	3.49 ± 1.06	3.55 ± 1.04	0.29	0.78
Hypertension (*n*)	11	12	0.06	0.81
Diabetes (*n*)	10	8	0.27	0.60
Hyperlipidemia (*n*)	9	11	0.25	0.62
Smoking (*n*)	11	10	0.06	0.81
Drinking (*n*)	23	20	0.37	0.55

**Table 2:** Comparison of complication rates.

Group	Deep venous hematoma of lower extremity	Rash	Tumor cell proliferation and metastasis	Total incidence rates
Experimental group	2	2	1	10%
Control group	5	6	4	30%
*X* ^2^				6.25
*P*				0.01

## Data Availability

The datasets used and/or analyzed during the current study are available from the corresponding author on reasonable request.
